# Antioxidative and antiatherogenic effects of flaxseed, α-tocopherol and their combination in diabetic hamsters fed with a high-fat diet

**DOI:** 10.3892/etm.2014.2102

**Published:** 2014-12-03

**Authors:** RALUCA ECATERINA HALIGA, VERONICA MOCANU, MAGDA BADESCU

**Affiliations:** Department of Pathophysiology, Grigore T. Popa University of Medicine and Pharmacy, Iaşi 700115, Romania

**Keywords:** diabetes mellitus, atherosclerosis, oxidative stress, golden Syrian hamster, flaxseed, vitamin E

## Abstract

Oxidative stress has previously been shown to play a role in the pathogenesis of diabetes mellitus (DM) and its complications. In the present study, the effects of supplementation with dietary antioxidants, flaxseed and α-tocopherol were investigated in diabetic golden Syrian hamsters fed with a high-fat diet. Thirty-five golden Syrian hamsters were randomly divided into a control group (C) and four diabetic groups (DM, DM + flax, DM + E and DM + Flax + E). The hamsters received four different diets for a 20-week period, as follows: i) Groups C and DM received a high-fat diet (40% energy as fat), deficient in α-linolenic acid (ALA); ii) the DM + Flax group received a high-fat diet enriched with ground flaxseed 15 g/100 g of food, rich in ALA; iii) the DM + E group received a high-fat diet enriched with vitamin E, 40 mg α-tocopherol/100 g of food; and iv) the DM + Flax + E group received a high-fat diet enriched with flaxseed and vitamin E. The results of serum lipid and oxidative stress analysis suggested that the antiatherogenic effect of flaxseed, α-tocopherol and their combination added to a high-fat diet in diabetic hamsters was based primarily on their antioxidative role, demonstrated by decreased serum lipid peroxidation and increased liver glutathione content. Improvements of serum glucose and non-high-density lipoprotein cholesterol (HDL-C) levels were observed and may have contributed to the prevention of diabetic macroangiopathy evidenced in the histopathological examination. The antioxidant effect of flaxseed was similar to that of α-tocopherol in diabetic hamsters fed a high-fat diet and combined supplementation did not appear to bring more benefits than flaxseed alone. Moreover, the high dose of ground flaxseed alone may have a better cardioprotective effect than α-tocopherol in diabetic hamsters by reducing total cholesterol and non-HDL-C levels and increasing HDL-C levels.

## Introduction

Oxidative stress is considered to be significant in the pathogenesis of diabetes-induced cardiovascular disease (CVD), which is associated with an abnormal blood lipid profile, insulin resistance and metabolic syndrome (1). Oxidative stress occurs due to a disturbance of the balance between antioxidant defense mechanisms and the levels of reactive oxygen species (ROS) (2,3). Numerous studies have identified significant alterations in plasma antioxidant vitamins (including vitamins C, E and A), antioxidant enzyme systems [superoxide dismutase (SOD), catalase (CAT) and glutathione peroxidase (GSH-Px)] and in lipid peroxidation in diabetes (4,5). In chronic diabetes mellitus (DM), the stability and reactive capacity of antioxidants seriously affect the long-term complications caused by oxidative stress (6,7). Antioxidants have been shown to reduce complications in DM by preventing free radical-mediated damage (4,8).

Dietary supplementation with antioxidants, including vitamins and phenolic compounds obtained from plants, may help to maintain a desirable pro-oxidative/antioxidative balance (9,10). A variety of dietary sources are presently of considerable interest due to their potential health benefits in relation to numerous diseases, including diabetic disorders (11,12). Flaxseed (also known as linseed and *Linum usitatissimum*), an edible oil seed/grain from a traditional arable crop, has been acknowledged as a functional food (13), and is the focus of considerable attention due to its unique nutrient components and its potential to prevent CVD (14). In addition of being one of the richest plant sources of α-linolenic acid (ALA; ~22% of whole flaxseed), flaxseed is an essential source of lignans (in particular, secoisolariciresinol diglucoside, SDG) (15). SDG has demonstrated extreme radical scavenging activity, thereby protecting polyunsaturated fatty acids from oxidation (16–18). Despite the beneficial effects of SDG, flaxseed consumption has been found to significantly reduce α- and γ-tocopherol concentrations in rats (19) and only vitamin E supplementation was able to restore the plasma concentrations (20).

α-tocopherol supplementation has previously been demonstrated to be beneficial in increasing the levels of antioxidant enzymes such as SOD and GSH-Px, and of reduced GSH in diabetes (21–23); however, little is known about the effect of adding vitamin E to a flaxseed-enriched diet on oxidative stress and aortic atherosclerotic lesions in diabetes.

In the present study, the effects of dietary flaxseed, α-tocopherol and their combination were investigated on atherosclerotic progression in diabetic hamsters fed a high-fat diet by examining serum lipid concentrations, oxidative stress markers, aortic cholesterol content and aortic histological aspects.

## Materials and methods

### Animals

A total of 35 male Golden Syrian hamsters were used in the study. The hamsters were purchased from the Cantacuzino National Institute for Research and Development in Microbiology and Immunology (Bucharest, Romania). This study was approved by the Laboratory Animal Care Committee of Grigore T. Popa University of Medicine and Pharmacy (Iaşi, Romania), and the hamsters were maintained in accordance with the general guidelines for the care and use of laboratory animals recommended by the Council of European Communities (24).

The hamsters were caged singly and kept in standard laboratory conditions with a controlled temperature (20±2°C) and a 12 h light/12 h dark cycle. Diabetes was induced in the hamsters using streptozotocin (STZ; catalog no. S0130; Sigma-Aldrich, St. Louis, MO, USA) (25). STZ, at a dose of 50 mg/kg body weight, freshly solved in citrate buffer (50 mM, pH 4.5), was administered intraperitoneally, as a single dose in the morning, following a night of fasting. Citrate buffer (50 mM) was prepared from sodium citrate and citric acid (S.C. Chemical Company, Iaşi, Romania) dissolved in distilled water, with adjustment of the pH to 4.5. The control group (C) received an equivalent quantity of citrate buffer (50 mM), administered intraperitoneally. All animals having a blood glucose level >126 mg/dl (7 mmol/l) were considered to be diabetic.

### Grouping and diets

Each hamster received 15 g food/day and tap water *ad libitum*. The animals were randomly divided into a control group (C) and four diabetic groups (DM, DM + flax, DM + E and DM + Flax + E). The hamsters received four different diets for a 20-week period, as follows: i) Groups C and DM received a high-fat diet (40% energy as fat), that was deficient in ALA; ii) the DM + Flax group received a high-fat diet enriched with ground flaxseed (Linum usitatissimum; 15/100 g of food), that was rich in ALA; Flaxseed of the Olin variety was provided by the Department of Phytotechny of the Faculty of Agronomy (Iaşi, Romania). iii) the DM + E group received a high-fat diet enriched with vitamin E (40 mg α-tocopherol/100 g of food; Sigma-Aldrich); and iv) the DM + Flax + E group received a high-fat diet enriched with a combination of flaxseed and vitamin E. All four diets had similar carbohydrate, total fiber, protein and fat contents (Table I).

### Animal necropsy and processing of samples

At the end of the experiment, the animals were sacrificed by cardiac puncture under ketamine anesthesia (100 mg/kg body weight). Blood samples were collected without anticoagulant. Aliquots of serum were frozen and kept at −80°C for subsequent analysis. The liver was immediately removed, rinsed with ice-cold saline, placed in a sealed container, homogenized for biochemical analysis and stored at −20°C until analyzed. The aortas were dissected, rinsed with cold saline and preserved in a phosphate buffer (pH 7.2).

### Serum glucose

Serum glucose was measured by enzymatic colorimetric methods on a Tecan microplate reader (Tecan SunriseTM Touchscreen, Männedorf, Switzerland) using the AD1A716 commercially available kits (Audit Diagnostics, Cork, Ireland).

### Serum lipid profile

Serum total cholesterol (TC), high-density lipoprotein cholesterol (HDL-C) and triglyceride (TG) levels were measured by enzymatic colorimetric methods on a Tecan microplate reader using the AD1A704, AD1A602 and AD1A306 commercially available kits (Audit Diagnostics). Non-HDL-C levels were calculated by subtracting the level of HDL-C from that of TC.

### Evaluation of cholesterol content in the aorta

The aortas of the hamsters in each group were removed. A section of the aortic arch of each animal was soaked in a 10% (v/v) formal saline solution and was stored on ice prior to being stained and fixed. The remainder of the aorta was soaked in phosphate-buffered saline (PBS) and homogenized for biochemical analysis. The lipid content was extracted by treatment with chloroform and methanol followed by centrifugation (26). The extracted lipid was dissolved in ethanol and measured using a AD1A704 cholesterol assay kit (Audit Diagnostics) utilizing absorbance spectrophotometry (Microlab 300, Vital Scientific, Spankeren, Netherlands) at 500 nm wavelength, and the amount quantified as μg/mg wet tissue.

### Parameters of oxidative stress

Serum and liver thiobarbituric acid reactive substances (TBARS) are indices of lipid peroxidation and oxidative stress. TBARS were determined using the method described by Phelps and Harris (27). The quantity of the TBARS was measured using a Tecan microplate reader at a wavelength of 540 nm.

Liver levels of reduced GSH were determined by an enzymatic reaction, based on the oxidation of GSH by 5,5′-dithiobis(2-nitrobenzoic acid) (DTNB), in the presence of GSH reductase and methylenetetrahydrofolate reductase, monitored at a wavelength of 405 nm (28). Liver SOD levels were determined using the method described by Minami and Yoshikawa (29).

### Morphological study of the aorta

For evaluation of aortic atherosclerotic lesions by light microscopy, frozen sections of 10 μm thickness were taken from the region of the proximal aorta. The extent of atherosclerosis was visually assessed after cutting the frozen sections at a size of 8–10 mm, fixing them in formalin, briefly washing them with running tap water for 1–10 mins and rinsing with 60% isopropanol prior to staining the sections with Oil Red O (3 mg/ml Oil Red O in 60% acetone and 40% water; Sigma-Aldrich). The samples were then counterstained with hematoxylin and the samples were examined under a light microscope (Olympus BX40, Olympus, Tokyo, Japan).

### Statistical analysis

Data are expressed as the mean ± standard deviation (SD). Univariate statistical analysis was performed using the Student’s t-test and Bonferroni’s multiple comparison test (Statistical Software Package SPSS^®^, version 13, SPSS Inc., Chicago, IL, USA).

## Results

### Serum glucose

The addition of flaxseed or/and vitamin E to the high-fat diet led to significant reductions of serum glucose levels compared with those in the DM group (Table II).

### Serum lipid profile parameters

Diabetes resulted in significant increases in the serum concentrations of TC, TG and non-HDL-C, and a significant reduction of HDL-C concentrations compared with those in the control group. Flaxseed supplementation significantly decreased serum TC and non-HDL-C levels and increased HDL-C levels (Table II) compared with those in the unsupplemented DM group. The addition of vitamin E to the flaxseed-rich diet significantly decreased TC, non-HDL-C and TG levels but did not improved the HDL-C level in diabetic hamsters.

### Cholesterol content of the aorta

Aortic cholesterol contents were significantly increased in the DM group fed with a standard diet compared with those in the control group (Table II). Flaxseed or/and vitamin E supplementation of the diet significantly decreased the aortic cholesterol content in the hamsters with DM (Table II).

### Parameters of oxidative stress

The main findings are summarized in Table III. Serum and liver TBARS, as indices of lipid peroxidation, were significantly increased in the DM group compared with those in the control group, while the addition of flaxseed or a combination of flaxseed and α-tocopherol to the high-fat diet of the hamsters with DM significantly decreased these two markers compared with those in the unsupplemented DM group. Liver GSH levels were significantly diminished in the DM group compared with those in the control group. Flaxseed, α-tocopherol and their combination added to the high-fat diet significantly increased the liver GSH levels in the diabetic hamsters. The increased in liver GSH content was significantly higher in the DM + Flax + E group compared with that in the DM + Flax group. No significant differences of SOD activity in the liver were identified between groups.

### Histological changes in aortic tissues

#### Control group

The histologic examination of aortal fragments with O-Rd staining revealed discrete thickening of the aortic intimal layer (Fig. 1A).

#### Diabetic groups

The histologic examination of aortic fragments with O-Rd staining from diabetic hamsters revealed morphologic changes specific to diabetic macroangiopathy (Fig. 1B). Intimal thickening, endothelial discontinuities, lipid drops in the subintimal space, and alterations to the middle layer of the arterial wall were observed. The addition of flaxseed and/or vitamin E to the high-fat diet in diabetic hamsters improved the histological aspects of aortic atherosclerosis described in the diabetic hamsters fed an unsupplemented diet. The aortal tissue in the supplemented groups was characterized by slightly swollen endothelium, with moderate intimal thickening and moderate lipid infiltration of the intima (Fig. 2).

## Discussion

In DM, oxidative stress occurs, primarily due to the increased production of oxygen free radicals and/or a reduction in the antioxidant defense. Numerous studies have demonstrated that an increase in oxidative stress is implicated in the pathogenesis and progression of diabetic vascular lesions (1,4,6).

In the present study, the antioxidative and antiatherosclerotic effects of supplementation with flaxseed (15 g *Linum usitatissimum*/100 g food), α-tocopherol (40 mg α-tocopherol/100 g food), and their combination were investigated in an animal model that replicates human atherosclerotic lesions. Golden Syrian hamsters appear more predisposed to develop atherosclerotic lesions than rats (30), and present many similarities with the lipoprotein metabolism in humans (31). In hamsters, a 15% flaxseed-supplemented diet is similar in energetic load to the 40 g/day dosage used in human trials. In humans, high doses of 40–50 g flaxseed/day, which corresponds to ~10% of total energy intake have been used in trials (32).

In the present study, it was hypothesized that adding vitamin E to the flaxseed diet would lead to improved results for oxidative stress and the prevention of atherosclerotic lesions as there is evidence that the consumption of flaxseed reduces vitamin E (19), and only vitamin E supplementation is able to restore the plasma concentration (20).

The present study demonstrated that all three diets (flaxseed, α-tocopherol or their combination) had an antiatherogenic effect in diabetic hamsters, suggested by the prevention of histological lesions (reduced intimal lipid infiltration and discrete alterations to the middle layer of the arterial wall) and by the decreased aortic cholesterol content in supplemented diabetic hamsters compared with those in the unsupplemented diabetic group. The antiatherogenic mechanism of the diets used in our experiment may be associated with changes in metabolic parameters, particularly in glucose concentrations and the lipid profile, and oxidative stress.

Flaxseed, α-tocopherol, and the combination of flaxseed and α-tocopherol added to the high-fat diet resulted in similar reductions in serum lipid peroxidation in the diabetic hamsters. Liver lipid peroxidation was significantly diminished by supplementation of the diet by flaxseed alone or in combination with α-tocopherol, but not by α-tocopherol supplementation alone. Moreover, all three diets increased the liver GSH content and the highest concentrations were obtained with the combined diet.

These results suggest that the higher antioxidant effects of flaxseed plus vitamin E are due to their synergic antioxidant actions. Flaxseed is the richest source of the lignan SDG. SDG isolated from flaxseed has oxygen radical-scavenging properties that have been demonstrated *in vitro* by direct hydroxyl radical-scavenging activity (18) or by inhibition of lipid peroxidation (16). Vitamin E is known as a major antioxidant in the cellular antioxidant defense system, which acts by interrupting the propagation of free radical chain reactions. The effect of vitamin E against the prooxidant status associated with DM has been demonstrated by the suppression of diabetes-induced increases in ROS and diminishment of lipid peroxidation (33,34). The synergistic effect of flaxseed oil and vitamin E on oxidative stress has also been observed by Deng *et al* (35) in male Wistar rats fed a high-fat diet.

Similar to the findings of previous studies (36), the diabetic hamsters had higher serum concentrations of serum glucose, TC, TG and non-HDL-C, and lower HDL-C concentrations compared with the control group. The addition of flaxseed, α-tocopherol or their combination to the high-fat diet reduced serum concentrations of glucose, TC and non-HDL in diabetic male hamsters (37,38). The hypocholesterolemic effects of flaxseed may be attributed to ALA, lignans (SDG) or the fiber content (39). In agreement with other studies (40), vitamin E significantly reduced serum TG levels in diabetic hamsters fed an atherogenic diet. In the present study, the addition of vitamin E alone or in combination with flaxseed to the high-fat diet resulted in lower serum concentrations of TC, non-HDL and TG but failed to correct the HDL-C concentrations in diabetic hamsters. Another study has reported that in hamsters with experimental STZ-induced DM fed high a saturated fat and cholesterol diet, supplementation with α-tocopherol increased TC and did not change HDL-C (40).

The results of the present study suggest that the antiatherogenic effect of flaxseed, α-tocopherol and their combination added to a high-fat diet in diabetic hamsters is based primarily on the antioxidative role of these components. The improvement of serum glucose and non-HDL were evident and could contribute to the prevention of diabetic macroangiopathy. The antioxidant effect of flaxseed was similar to that of α-tocopherol in diabetic hamsters fed a high-fat diet and the combined diet (Flax + E) did not seem to confer more benefits than flaxseed alone. Moreover, the high dose of ground flaxseed alone may have a better cardioprotective effect than α-tocopherol in diabetic hamsters due to the reduction of TC and non-HDL levels and increase in HDL-C levels.

Oxidative stress has been proposed as a pathogenic mechanism of diabetic macrovascular complications, and dietary strategies that ameliorate oxidative stress may represent a promising approach to the prevention of atherosclerosis.

The flaxseed-enriched diet may regulate the generation of reactive oxygen species and the metabolism of glucose and lipids, and could consequently play a role in the prevention of major cardiovascular complications in diabetic states. Ground flaxseed combined with α-tocopherol does not appear to confer a clear advantage compared with flaxseed alone in the reduction of oxidative stress and vascular lesion formation in experimental diabetes.

## Figures and Tables

**Figure 1:** Images of the aorta. (A) Aortal tissue from the control group fed with a high-fat diet (Oil Red O staining; magnification, ×20). Moderate thickening of the aortic intimal layer (arrows) is present. (B) Aortal tissue from the diabetes mellitus group fed with a high-fat diet (Oil Red O staining; magnification, ×40). A thickened intima, discontinuous endothelium, a few macrophages in the intimal space, lesions in the middle arterial layer, and pronounced infiltration of the intima with lipid vesicles (arrows) is present.

**Figure 2:** Images of the aorta. (A) Diabetes mellitus (DM) + flaxseed (Flax) group (Oil Red O staining; magnification, ×20). Moderate intimal thickening, endothelium with swollen cells, and moderate infiltration with lipid microvesicles in the intima and internal third of the media (arrows) were observed. (B) DM + Flax + vitamin E (Oil Red O staining; magnification, ×40). The endothelium is slightly swollen with infrequent areas of discontinuity, and a thickened intima with the rare presence of lipid drops (arrow), and moderate structural disorganization of elastic fibers in the middle layer of the vessel wall.

**Table I:** Composition of the diets.

Ingredients	High-fat diet (40% of energy as fat)	High-fat diet supplemented with flaxseed	High-fat diet supplemented with vitamin E	High-fat diet supplemented with flaxseed and vitamin E
Carbohydrates	330	330	330	330
Fiber	110	110	110	110
Proteins	240	240	240	240
Lipids	160	160	160	160
Saturated^a^	96	96	96	96
Monounsaturated	7	7	7	7
Polyunsaturated	57	57	57	57
n-6 PUFA (sunflower oil)	57	23	57	23
n-3 PUFA (flaxseed^b^)	-	34	-	34
Choline	3	3	3	3
Vitamin A (IU)	200000	200000	200000	200000
Vitamin C	1	1	1	1
Vitamin D (IU)	10000	10000	10000	10000
Vitamin E	0.05	0.05	0.4	0.4
Calcium	6.2	6.2	6.2	6.2
Phosphate	3.9	3.9	3.9	3.9
Potassium bicarbonate	20	20	20	20

Quantities are g/kg diet, unless otherwise indicated. PUFA, polyunsaturated fatty acid.

a Hydrogenated coconut oil.

b Flaxseeds (*Linum usitatissimum*) of the Olin variety, provided by the Department of Phytotechny, Faculty of Agronomy Iaşi. The composition of the flaxseeds was: 40.2% oil (55.6% linolenic acid) and 19.5% proteins.

**Table II:** Serum glucose, serum lipid profile and aortal cholesterol content in the study groups.

Parameter	C	DM	DM + Flax	DM + E	DM + Flax + E
Serum					
Glucose (mg/dl)	62±7	362±99^a^	139±43^a^,^b^	143±43^a^,^b^	163±47^a^,^b^
TC (mg/dl)	232±7	275±13^a^	206±5^a^,^b^	146±26^a^,^b^	164±1^a^–^c^
TG (mg/dl)	217±10	331±31^a^	313±12^a^	159±30^a^,^b^	94±17^a^–^c^
HDL-C (mg/dl)	78±7	43±5^a^	81±10^b^	46±7^a^	34±5^a^
Non-HDL	154±5	231±13^a^	125±11^a^,^b^	100±30^a^,^b^	130±12^b^
Aortal cholesterol (μg/mg wet tissue)	3.6±1.4	4.8±1.7^a^	4.1±1.9^b^	4.0±0.9^b^	4.2±1.5^b^

Values are presented as the means ± standard deviation; n=7 in each group. TC, total cholesterol; TG, triglycerides; HDL-C, high-density lipoprotein cholesterol; C, control; DM, diabetes mellitus; Flax, flaxseed; E, vitamin E.

a P<0.05 compared with group C.

b P<0.05 compared with the DM group.

c P<0.05 compared with the DM + Flax group.

**Table III:** Oxidative stress parameters in the study groups.

Parameters	C	DM	DM + Flax	DM + E	DM + Flax + E
Serum TBARS (nmol/ml ser)	1.6±0.5	4.3±1.4^a^	1.6±0.5^b^	2.6±1.0^a^,^b^	2.5±0.9^b^
Liver TBARS (nmol/mg prot)	12.0±1.2	14.5±2.3^a^	11.9±2.2^b^	15.4±0.9^a^	12.1±1.8^b^
Liver GSH (μM/mg prot)	17.3±5.6	10.6±2.1^a^	15.5±3.3^b^	20.7±4.4^b^	33.6±3.9^a^–^c^
Liver SOD (U/mg prot)	12.1±0.8	11.3±0.7	12.4±1.6	12.9±0.9^b^	12.5±0.9

Values are means ± standard deviation; n=7 in each group. TBARS, thiobarbituric acid reactive substances; GSH, glutathione; SOD, superoxide dismutase; C, control; DM, diabetes mellitus; Flax, flaxseed; E, vitamin E.

a P<0.05 compared with group C.

b P<0.05 compared with the DM group.

c P<0.05 compared with the DM + Flax group.
